The article "Metastatic Cervical Cancer: A Case That Recalls the Importance of a Multidisciplinary Approach" was published in 2023. Journal: Cureus.

# Metastatic Cervical Cancer: A Case That Recalls the Importance of a Multidisciplinary Approach

**DOI:** 10.7759/cureus.48626

**Published:** 2023-11-10

**Authors:** Ana R Teixeira, Miguel H Abreu

**Affiliations:** 1 Oncology, Instituto Português de Oncologia, Porto, PRT

**Keywords:** multidisciplinary health team, neoplasm metastasis, locoregional neoplasm recurrence, cervical cancer, gynecologic neoplasms

## Abstract

Cervical cancer is one of the most common neoplasms in women. Usually, this cancer is only symptomatic in advanced stages and is associated with a poor prognosis. We present the case of a 34-year-old woman with localized cervical cancer at diagnosis treated with surgery in 2011. Six years later, she presented recurrent disease with vaginal, pelvic, and lung metastases. Since then, the patient completed three lines of chemotherapy and a line of immunotherapy, and she was submitted to external radiotherapy and orthopedic surgery. Currently, the patient keeps regular follow-ups and maintains a good performance status. The treatment of recurrent cervical cancer remains a challenge, and the prognosis is poor. This case emphasized the importance of multidisciplinary discussion towards cases of locally advanced or metastatic cervical cancer, which may change this paradigm.

## Introduction

Worldwide, cervical cancer (CC) is the fourth most common cancer and the third cause of cancer-related death among women [1]. The incidence of CC has decreased over the decades, mostly in developed countries, due to screening for preneoplastic lesions in cervical cytology (Papanicolaou test), detection of human papillomavirus (HPV), and HPV prophylactic vaccination [2]. The most important etiological factor for CC is HPV infection (mostly HPV 16 and 18), which is more prevalent in young and child-bearing age women, with a peak incidence in the fourth decade [2,3]. In contrast, CC remains an important health problem in low-income and middle-income countries, with the highest morbidity and mortality [2]. This is probably related to the highest HPV incidence and later cancer diagnosis [2].

Usually, CC is only symptomatic in advanced stages, causing abnormal vaginal bleeding, discharge, pelvic pain, and dyspareunia [3]. Five-year overall survival (OS) in locally advanced and metastatic settings is approximately 65% and 17%, respectively [4].

## Case presentation

We present the case of a 34-year-old woman without any relevant medical history who was diagnosed with an early-stage usual-type poorly differentiated cervical adenocarcinoma with PD-L1 positivity (based on combined positive score). She underwent a Wertheim-Meigs operation in 2011, and the postoperative staging was pT1b1N0.

Six years later, a physical examination revealed a lesion measuring one centimeter on the right side of the vaginal cup. Histology confirmed adenocarcinoma metastasis, and re-staging imaging exams revealed two pelvic lesions, an enlarged internal iliac lymph node, and a lung lesion. She began systemic treatment with chemotherapy (cisplatin plus paclitaxel) in addition to bevacizumab, an anti-angiogenic monoclonal antibody. After six cycles of treatment, she kept bevacizumab-based maintenance therapy every 21 days for two years. 

In April 2020, the patient presented vaginal progressive disease. As she only had local progression, after discussion in a multidisciplinary tumor board, she was submitted to pelvic radiotherapy (45 Gy, delivered in 25 fractions and 1.8 Gy/day) and an additional boost to the vaginal lesion (20 Gy, delivered in 2 Gy/day). She completed radiotherapy with good tolerance.

A hepatic lesion and a lesion in the right femur appeared three months after the radiotherapy was finished (Figure 1A), along with an increase in serum squamous cell carcinoma antigen (SCC Ag) (Figure 2). The patient was started on a chemotherapy treatment with carboplatin and paclitaxel. Due to hematological toxicity, chemotherapy was stopped after five cycles. At that point, she had a hepatic complete response and a femur-stable disease (Figure 1B).

**Figure 1:** Disease evolution on 18fluorodeoxyglucose positron emission tomography (18FDG-PET) images A) Blue arrows demonstrate liver and right femur metastases (December 2020); B) Absence of 18FDG uptake, indicating complete response (November 2021); C) Blue arrows demonstrate right femur and ipsilateral inguinal and external iliac lymph nodes metastases (October 2022); D) Worsening 18FDG uptake of the right femur and ipsilateral inguinal and external iliac lymph nodes (January 2023); E) Minor 18FDG uptake by right hip indicating disease persistence or inflammatory disease (September 2023)

**Figure 2:** Evolution of serum squamous cell carcinoma antigen marker along patient's metastatic disease ChT - chemotherapy; IT - immunotherapy; RT - radiotherapy; SCC Ag - Squamous cell carcinoma antigen

After a new discussion in a multidisciplinary tumor board, it was decided to perform an orthopedic excision surgery. A proximal femoral excision and right hip reconstruction using a modular mega prosthesis were performed in October 2021 (Figure 3) without any complications, and the patient had an excellent functional recovery.

**Figure 3:** The right hip plain radiograph after orthopedic surgery Blue arrows indicate a modular mega prosthesis in the right hip

A year later, the surveillance 18-fluorodeoxyglucose positron emission tomography (18FDG-PET) revealed ipsilateral inguinal and external iliac lymph nodes, as well as a right femur disease recurrence (Figure 1C). As the patient maintained a good performance status, she started immunotherapy with cemiplimab, an immune checkpoint inhibitor targeting the programmed cell death 1 (PD-1) receptor. However, after three cycles, there was a new recurrence in the right femur and ipsilateral inguinal and external iliac lymph nodes and de novo right lung small nodules (Figure 1D). The patient started chemotherapy (carboplatin plus paclitaxel), but after the fourth cycle developed a platinum hypersensitivity reaction, and the treatment was suspended. After a new 18FDG-PET showing femoral disease persistence, the patient underwent local palliative radiotherapy (30 Gy, delivered in 10 fractions and 3 Gy/day) with good tolerance.

The patient is currently being monitored and maintains a satisfactory performance status six years following the recurrence of cervical cancer (Figure 1E).

## Discussion

There are three categories of epithelial tumors of the cervix: squamous (70-80%), adenocarcinoma (10-25%) and other epithelial tumors [3]. It might be important to distinguish between HPV-associated or HPV-independent adenocarcinoma, as the last one is more common in older patients and is associated with a worse prognosis [5]. 

Recurrent CC is defined as local re-growth or local or distant metastasis at least six months after the primary lesion has regressed [6]. The most frequent sites of recurrence are local (vaginal) or regional [6]. Around 30% of CC patients will have recurrent disease (27% following primary surgery and 32% after chemoradiotherapy), and the prognosis remains poor in this setting, with an estimated overall survival (OS) of 13-17 months and a five-year OS rate of 17% in metastatic/recurrent disease [4,6].

In 2014, the GOG-240 trial provided evidence that the addition of bevacizumab to platinum-based chemotherapy in patients with recurrent, persistent, or metastatic CC was associated with longer median OS, so this became the standard first-line treatment in these settings [4,7]. More recently, it was proven the benefit of immunotherapy in locally advanced and metastatic CC [4]. For cancers with PD-L1 CPS ≥1, the first-line treatment should be platinum-based chemotherapy in combination with bevacizumab and pembrolizumab, an immune checkpoint inhibitor [4]. Regarding our case report, which is prior to this evidence, the patient only received immunotherapy monotherapy after disease progression, which is in line with European Society for Medical Oncology (ESMO) recommendations [4].

Radiotherapy also plays a role in the management of locally advanced or metastatic CC [8]. If there is locally advanced or limited distant metastatic disease, curative intent treatment with definitive platinum-based chemoradiotherapy or brachytherapy should be considered [8]. Even in patients with disseminated disease, palliative radiotherapy (usually a fractionated course) could be offered to control symptoms such as bleeding or pain [8].

The management of recurrent CC should always be discussed in a multidisciplinary team involving gynecologists, radiation oncologists, medical oncologists, radiologists, pathologists, urologists, and plastic surgeons [8]. The treatment must be individualized because it will differ depending on previous treatments and recurrence location and extent [6].

## Conclusions

In conclusion, recurrent or metastatic cervical cancer is associated with a poor prognosis. Maybe careful patient selection, early detection of recurrent/ metastatic disease, and multidisciplinary team discussion could be the key to tailoring the choice of salvage treatment and improving OS in these patients. The existence of a well-established multidisciplinary group for the discussion of more complex problems may also allow patients to keep their quality of life, as previously described, which is crucial in the advanced disease settings of any cancer type. 
